# Upregulation of miR-29c-3p Hinders Melanoma Progression by Inhibiting CDCA4 Expression

This article has been retracted.

**DOI:** 10.1155/2021/7065963

**Published:** 2021-08-28

**Authors:** Jiazheng Liu, Guilu Tao, Cundi Zhong, Xiao Liu

**Affiliations:** ^1^Department of Laboratory, Second Affiliated Hospital of Dalian Medical University, Dalian, Liaoning Province, China; ^2^Department of Wound Repairment, Second Affiliated Hospital of Dalian Medical University, Dalian, Liaoning Province, China

## Abstract

**Objective:**

To investigate the expression and regulation mechanism of miR-29c-3p and cell division cycle associated 4 (CDCA4) in melanoma (MM). *Data and Methods*. Fifty-nine patients with MM admitted to our hospital were enrolled as the MM group. They were followed up for 3 years to analyze the prognostic factors; meanwhile, 51 healthy subjects were allocated into a normal group. MM cell lines (M21 and C8161) were transfected with miR-29c-3p-mimics, miR-29c-3p-inhibitor, miR-NC, si-CDCA4, and sh-CDCA4. The expression of miR-29c-3p, CDCA4, Bax, Caspase3, Bcl-2, N-cadherin, vimentin, and E-cadherin was quantified, and cell proliferation, migration, invasion, and apoptosis, as well as epithelial-mesenchymal transition (EMT), were determined.

**Results:**

Serum miR-29c-3p was lowly expressed and CDCA4 was highly expressed in the MM group. The area under the curve (AUC) of both for diagnosing MM was greater than 0.9. miR-29c-3p and CDCA4 were related to regional lymph node staging (N staging), distant metastasis (M staging), tumor diameter, and pathological differentiation. Low miR-29c-3p and high CDCA4 were associated with poor prognosis of MM. Overexpression of miR-29c-3p and suppression of CDCA4 hindered cell proliferation, migration, invasion, and expression of Bax, Caspase3, N-cadherin, and vimentin, but cell apoptosis and expression of Bcl-2 and E-cadherin were enhanced. Dual-luciferase reporter (DLR) assay confirmed the targeted relationship between miR-29c-3p and CDCA4. After miR-29c-3p-mimics+sh-CDCA4 was transfected into M21 and C8161 cells, the proliferation, invasion, and apoptosis were not different from those in the miR-NC group transfected with unrelated sequences.

**Conclusion:**

Overexpression of miR-29c-3p suppresses CDCA4 expression and decreases proliferation, migration, invasion, apoptosis, and EMT of MM cells, thus hindering MM progression.

## 1. Introduction

Melanoma (MM) is a prevalent malignant tumor in western countries with a highly heterogeneous prognosis in advanced patients and a rising incidence [1, 2]. According to epidemiological statistics, the 10-year survival is less than 30%, with 232,000 new cases and 55,000 deaths worldwide [3, 4]. The treatment mostly depends on clinical stages, tumor diameter, gene mutation, and other pathological data. Resection operation is the preferred choice for early-stage patients, and interferon-*α*- (INF-*α*-) based adjuvant therapy and systemic therapy were generally applied to middle- and advanced-stage patients, respectively. However, those treatment regimens are more or less potentially dangerous [5]. Progression to advanced MM leads to greatly reduced therapeutic effectiveness and high cost, and the best way to prevent the progression is early diagnosis [6]. At present, the diagnosis of MM mainly relies on pathological biopsy and computer-assisted imaging techniques which have the limitations of low acceptability, high cost, and complicated operation [7]. Therefore, it is of great significance to find reliable, convenient, and cost-effective biological diagnostic indicators for prevention, early diagnosis, and treatment of MM.

MicroRNAs (miRNAs) regulate gene expression through a variety of biological mechanisms and have excellent pathological regulation functions in cancer cells and the tumor microenvironment [8–10]. The abnormal expression of miRNAs in the serum of MM patients provides a new insight for serum-based noninvasive diagnosis of MM, and a number of miRNAs have been reported to be available for the early diagnosis of this disease [11, 12]. miR-29c-3p is a member of the miRNA family and miR-29 family. miR-29a/b functions as a cytokine signal transducer in the IFN-*γ*-related MM regulation mechanism, while miR-29c-3p is involved in MM progression by mediating methylation of relevant genes, which is valuable for evaluating the prognosis of the patients [13, 14]. Cell division cycle associated 4 (CDCA4) is a functional protein that interferes with the cell cycle by participating in the transcriptional activation of transcription factor E2F, and its expression in cancer cells is capable of regulating cell growth and DNA synthesis [15]. As a direct target for miR-15a, CDCA4 affects growth and invasion of mouse MM cells, playing an essential role in the regulatory mechanism of MM [16].

In this study, online target gene prediction software (http://www.targetscan.org/vert_72/) demonstrated that CDCA4 shared target loci with miR-29c-3p, so we speculated that miR-29c-3p affected the biological function of MM cells by targeting CDCA4. We aimed to investigate the expression and regulation mechanism of miR-29c-3p and cell division cycle associated 4 (CDCA4) in melanoma (MM).

## 2. Data and Methods

### 2.1. Clinical Data

Fifty-nine patients (33 males and 26 females, average age: 58.65 ± 7.33 years) with MM who were admitted to our hospital from March 2014 to March 2016 being enrolled as the MM group. Another 51 healthy individuals (29 males and 22 females, average age: 58.43 ± 7.18 years) were enrolled. There was no significant difference in sex and age between the two groups (*P* > 0.05), indicating a comparability.

### 2.2. Inclusion Criteria

Patients diagnosed with MM by pathology or laboratory indicators [17] and meeting tumor-node-metastasis (TNM) staging criteria [18], patients treated for the first time, and patients who received no drugs that affected the indicators of this study within half a year were included. Exclusion criteria are as follows: patients with other malignant tumors, organ dysfunction, other skin diseases, or infectious and autoimmune diseases. All patients and their families agreed to participate in the study and signed the informed consent form. Hospital Ethics Committee approval was obtained.

### 2.3. Experimental Reagents and Materials

Human MM cell lines M21, MV3, C8161, and FM88 and normal skin cell line HFF (C0815, C0922, GD-C0038632A66388, GD-C0038632A67230, GD-C0038632A65580, Guandao Bioengineering Co., Ltd., Shanghai, China); Lipofectamine™ 2000 Kit (11668019, Woosen Biological Technology Co., Ltd., Hangzhou, Zhejiang, China); TransScript Green miRNA Two-Step qRT-PCR SuperMix and TransScript II Green Two-Step qRT-PCR SuperMix (abx098036, abx098035, QW Biotechnology Co., Ltd., Beijing, China); methyl thiazolyl tetrazolium (MTT) kit, radioimmunoprecipitation assay (RIPA), and TRIzol (111105-500, 9806S, KGA1201, Winter Song Boye Biotechnology Co. Ltd., Beijing, China); dual-luciferase reporter (DLR) assay kit, goat anti-rabbit (IgG) secondary antibody, fetal bovine serum (FBS), and enhanced chemiluminescence (ECL) developer (KFS303-TFX, WK363-BXY, QS071, GL1055-LIE, Baiao Laibo Technology Co., Ltd., Beijing, China); and phosphate buffer saline (PBS) and bicinchoninic acid (BCA) protein kit (120830, 120982, ChreaGen Biotechnology Co., Ltd., Beijing, China). CDCA4, Bax, Caspase3, Bcl-2, N-cadherin, vimentin, E-cadherin, and *β*-actin antibody (Kemin Biotechnology Co., Ltd., Shanghai, China); a polymerase chain reaction (PCR) instrument and flow cytometer (DLK0003730, DLK0002051, DERICA Biotechnology Co., Ltd., Beijing, China); an ultraviolet (UV) spectrophotometer (UV-1100, Peking University Care Industrial Park, Beijing, China); and primers (Beijing Future Biotechnology Co., Ltd.) were used.

### 2.4. Cell Culture, Passage, and Transfection

MM cell lines were cultured in Dulbecco's modified Eagle medium (DMEM) comprising 10% FBS at 37°C and 5% CO_2_. When reaching 85% confluence, the cells were digested with 25% Trypsin, then placed in the medium for continuous culture to complete passage, and, finally, transfected with miR-29c-3p-mimics (overexpression sequence) and miR-29c-3p-inhibitor (inhibition sequence), negative control miR (miR-NC), targeted inhibition of CDCA4 RNA (si-CDCA4), targeted overexpression of CDCA4 RNA (sh-CDCA4), and negative control RNA (si-NC) separately with a Lipofectamine™ 2000 kit.

### 2.5. Detection Methods

#### 2.5.1. Quantitative Real-Time PCR (qRT-PCR)

A TRIzol kit was employed to extract the total RNA from the collected serum and cells, and the purity and concentration were read with an UV spectrophotometer. Total RNA (5 *μ*g) was taken for reverse transcription, and 1 *μ*L of synthesized cDNA was served for amplification. The miR-29c-3p amplification system consists of the following: cDNA 1 *μ*L, upstream and downstream primers 0.4 *μ*L each, 2x TransTaq® Tip Green qPCR SuperMix 10 *μ*L, Passive Reference Dye (50x) 0.4 *μ*L, and finally made up to 20 *μ*L with ddH_2_O. Amplification conditions are as follows: PCR conditions: 94°C for 30 s, 40 cycles of 94°C for 5 s and 60°C for 30 s. The CDCA4 amplification system consists of the following: cDNA 1 *μ*L, upstream and downstream primers 0.4 *μ*L each, 2x TransScript® Tip Green qPCR SuperMix 10 *μ*L, Passive Reference Dye (50x) 0.4 *μ*L, and finally made up to 20 *μ*L with nuclease-free water. Amplification conditions consist of the following: 95°C for 30 s, 40 cycles of 95°C for 10 s and 60°C for 30 s. Each sample was provided with 3 repeated wells, and the test was conducted for 3 times. U6 and *β*-actin were served as an internal reference of miR-29c-3p and CDCA4, and 2^-△△ct^ was employed to analyze the data [19].

#### 2.5.2. Western Blot

Cultured cells were added with RIPA to extract the total protein, and the concentration was detected by BCA. The protein with a density of 4 *μ*g/*μ*L was separated by 12% sodium dodecylsulphate-polyacrylamide gel electrophoresis (SDS-PAGE) and grafted to a polyvinylidene difluoride (PVDF) membrane. The membrane was sealed with 5% defatted milk powder for 2 h, then added with CDCA4, Bax, Caspase3, Bcl-2, E-cadherin, N-cadherin, vimentin, and *β*-actin antibody (1 : 1000), and sealed overnight at 4°C. After removal of the *β*-actin antibody, a goat anti-rabbit secondary antibody (1 : 1000, HRP) was added; the membrane was incubated at 37°C for 1 h and rinsed with PBS for 3 times, 5 min each. Afterwards, the liquid was dried with filter paper. Development was carried out in a darkroom with an ECL developer. The protein bands were scanned to analyze the gray value in Quantity One software. Relative expression of protein = target protein band gray value/*β*-actin protein band gray value.

#### 2.5.3. MTT Assay for Cell Viability

MM cells harvested 24 hours after transfection (5∗10^3^ cells/well) were inoculated in 96-well plates at 37°C for 24, 48, and 72 hours, and 20 *μ*L MTT solution (5 *μ*g/mL) was added at each time point. After inoculating at 37°C for 4 h, 200 *μ*L dimethyl sulfoxide (DMSO) was added to each well. The optical density (OD) value was read by a spectrophotometer at the 490 nm wavelength.

#### 2.5.4. Wound Healing Assay for In Vitro Cell Migration

Cells diluted to 3∗10^5^ cells/mL were inoculated in 6-well plates. After reaching 85% confluence, a scratch was made artificially in monolayer cells using 200 *μ*L sterile pipette tips. The scratched cells were washed with PBS and cultured in a new medium. At 0 h (W0) and 24 h (W24) after scratching, cell migration was evaluated by a microscope though three scratches.

#### 2.5.5. Transwell for Cell Invasion

MM cells harvested 24 hours after transfection (3∗10^3^ cells/well) were inoculated in 24-well plates, then trypsinized and transferred to the apical chamber. RPMI 1640 solution (200 *μ*L) was added to the upper apical while RPMI 1640 (500 mL containing 10% FBS) to the basolateral chamber. After a 48 h culture at 37°C, substrates and cells in the apical chamber were removed. The membrane was washed 3 times with PBS, immobilized for 10 min with paraformaldehyde, washed another 3 times with double distilled water, and stained with 0.5% crystal violet after drying. Cell invasion was determined with a microscope.

#### 2.5.6. Flow Cytometry for Cell Apoptosis

Transfected cells were digested with 0.25% trypsin, washed twice with PBS, added with 100 *μ*L of binding buffer, and then prepared into 1∗10^6^/mL suspension. Annexin V-FITC and propidium iodide (PI) were added sequentially, and the suspension was incubated at room temperature in the dark for 5 min. Cell apoptosis was detected with a flow cytometer, and the test was repeated 3 times to take the average.

#### 2.5.7. DLR Assay

TargetScan7.2 predicted downstream target genes of miR-29c-3p. CDCA4 3′-untranslated region-wild type (3′UTR-Wt), CDCA4 3′UTR-mutant (Mut), miR-29c-3p-mimics, and miR-NC were transferred into M21 and C8161 cells using a Lipofectamine™ 2000 kit, and luciferase activity was determined in a DLR assay system.

### 2.6. Statistical Analysis

In our study, GraphPad 6 was employed for building graphs and processing data. Intergroup comparison was conducted with independent sample *t*-test and multigroup comparison with one-way analysis of variance (ANOVA) (denoted by *F*). The post hoc pairwise comparison was conducted with Fisher's least significant difference *t*-test, expression at multiple time points was analyzed with repeated measurement ANOVA (denoted by *F*), and the post hoc test was carried out with Bonferroni [20, 21]. The diagnostic value of miR-29c-3p and CDCA4 in MM was visualized with a receiver operating characteristic (ROC) curve [22]. Pearson's test identified the correlation of miR-29c-3p with CDCA4 in the serum, and the Cox analysis analyzed the independent prognostic factors of MM. A value of *P* < 0.05 indicated statistically significant difference [23–25].

## 3. Results

### 3.1. Expression and Diagnostic Value of Sera miR-29c-3p and CDCA4

The MM group exhibited remarkably lower serum miR-29c-3p and higher serum CDCA4 than the normal group (*P* < 0.05). The areas under the curve (AUC) of miR-29c-3p and CDCA4 for diagnosing MM were 0.912 and 0.939, respectively. Pearson's test revealed the negative correlation between the expressions of miR-29c-3p and CDCA4 (*r* = −0.671, *P* < 0.001). Both miR-29c-3p and CDCA4 were associated with regional lymph node staging (N staging), distant metastasis (M staging), tumor diameter, and pathological differentiation (*P* < 0.05), and miR-29c-3p is also closely correlated with tumor invasion staging (T staging) (*P* < 0.05) (see Figure 1 and Table 1).

### 3.2. Prognostic Value of Sera miR-29c-3p and CDCA4 in MM

All 59 patients with MM were followed up successfully for 3 years, and the 3-year overall survival (OS) was 27.12% (16/59). Among them, 16 dead patients were regarded as the poor prognosis group and 43 surviving patients as the good prognosis group. It turned out that patients in the poor prognosis group had remarkably lower serum miR-29c-3p and higher serum CDCA4 than those in the good prognosis group (*P* < 0.05). The AUC of miR-29c-3p and CDCA4 for predicting the poor prognosis of MM were 0.830 and 0.842, respectively. Low miR-29c-3p and high CDCA4 were correlated with lower OS. Cox regression revealed that TNM staging, tumor diameter, pathological differentiation, miR-29c-3p, and CDCA4 were independent prognostic factors of MM (see Figure 2 and Table 2).

### 3.3. Effects of miR-29c-3p on Biological Functions of MM Cells and Epithelial-Mesenchymal Transition- (EMT-) Related Proteins

miR-29c-3p showed suppressed expression in M21, MV3, C8161, and FM88 cells. After M21 and C8161 cells were transfected with miR-29c-3p-mimics, not only the miR-29c-3p-3p protein expression but also Bax, Caspase3, and E-cadherin expressions were elevated markedly, but the proliferation, migration, invasion, and protein expression of Bcl-2, N-cadherin, and vimentin were remarkably inhibited. However, opposite results were acquired when cells were transfected with miR-29c-3p-inhibitor (*P* < 0.05) (see Figure 3).

### 3.4. Effects of CDCA4 on Biological Functions of MM Cells and EMT-Related Proteins

CDCA4 showed elevated expression in M21, MV3, C8161, and FM88 cells. After M21 and C8161 cells were transfected with si-CDCA4, not only CDCA4 expression but also proliferation, migration, and invasion, as well as the Bcl-2, N-cadherin, and vimentin expressions, were inhibited, but the expressions of Bax, Caspase3, and E-cadherin were remarkably elevated. However, opposite results were acquired in cells transfected with sh-CDCA4 (*P* < 0.05) (see Figure 4).

### 3.5. Identification of miR-29c-3p Target Genes

Targeted binding loci between CDCA4 and miR-29c-3p were discovered by TargetScan7.2. Therefore, we conducted a DLR assay and found that the luciferase activity of pmirGLO-CDCA4-3′UTR-Wt decreased significantly after upregulating miR-29c-3p (*P* < 0.05), but that of pmirGLO-CDCA4-3′UTR-Mut showed no changes (*P* > 0.05). Western blot demonstrated that the expression of the CDCA4 protein in M21 and C8161 cells was remarkably suppressed after miR-29c-3p-mimics transfection (*P* < 0.05) (see Figure 5).

### 3.6. Cell Cotransfection

After transfecting miR-29c-3p-mimics+sh-CDCA4 and miR-29c-3p-inhibitor+si-CDCA4, M21 and C8161 cells showed no significant difference in proliferation, invasion, and expression of proteins compared with miR-NC (*P* > 0.05). However, compared with the cells transfected with miR-29c-3p-mimics, the proliferation, migration, and invasion and the expression of Bcl-2, N-cadherin, and vimentin proteins were remarkably enhanced, but the apoptosis and the expression of Bax, Caspase3, and E-cadherin proteins were remarkably inhibited. Compared with those transfected with the miR-29c-3p-inhibitor, all the results were reversed (*P* < 0.05) (see Figure 6).

## 4. Discussion

In this study, we found that miR-29c-3p hinders the progression of MM through the targeted inhibition of CDCA4. More and more scholars have shown great enthusiasm for the clinical value and regulation of miR-29c-3p and CDCA4 in human diseases; accordingly, numerous related researches emerged. For example, Licholai and Szczeklik stated that miR-29c-3p is a potential diagnostic indicator for patients with abdominal aortic aneurysm; it also inhibits the synthesis of the extracellular matrix by inhibiting related transcripts [26]. Besides, Chen et al. indicated that miR-29c-3p, a tumor suppressor, hinders invasion and migration of colon cancer cells by targeting the Pleckstrin homology-like domain family B member 2 (PHLDB2) [27]. In addition, according to Shi et al., silencing CDCA4 effectively inhibits the proliferation and accelerates the apoptosis of breast cancer cells [28].

The above findings remind us of the potential value of miR-29c-3p and CDCA4 in human diseases, so we explored their effects on MM in this study. It turned out that miR-29c-3p and CDCA4 showed low expression and high expression in the serum of MM patients, respectively, which made them available to distinguish the patients from healthy individuals. Therefore, we assessed the diagnostic value of miR-29c-3p and CDCA4 for MM. Surprisingly, the AUC of the two were 0.912 and 0.939, respectively, indicating their excellent diagnostic value for MM. We also analyzed the potential clinical value of miR-29c-3p and CDCA4. The results revealed that both were closely related to N staging, M staging, tumor diameter, and pathological differentiation, and miR-29c-3p was also related to T staging. Therefore, both miR-29c-3p and CDCA4 participate in the pathological process of MM and have a potential value in predicting pathological parameters of patients. We also found that low miR-29c-3p and high CDCA4 in serum were associated with poor prognosis and low 3-year OS of MM patients. Cox regression confirmed that both were independent prognostic factors of MM and so were TNM staging, tumor diameter, and pathological differentiation. In the study of Mirili, it was also pointed out that TNM staging, ulcer, and prognostic nutritional index (PNI) are independent predictors of OS of patients with MM [29], which indicates that PNI may also be a prognostic indicator of MM.

The above is our exploration on the potential clinical value of miR-29c-3p and CDCA4; next, the biological function analysis has been carried out. The expression of miR-29c-3p and CDCA4 in MM cell lines was consistent with that in the serum. We transfected M21 and C8161 cells with the most significant expression in cell lines. Cells transfected with miR-29c-3p-mimcs or si-CDCA4 showed not only lower proliferation, migration, and invasion but also higher apoptosis. However, opposite results were achieved in the cells transfected with the miR-29c-3p-inhibitor or sh-CDCA4. The above results suggested that overexpression of miR-29c-3p or knockdown of CDCA4 may play a role in hindering MM progression. In addition, the DLR assay showed that overexpressed miR-29c-3p remarkably reduced luciferase activity of pmirGLO-CDCA4-3′UTR-Wt, but it had no effect on pmirGLO-CDCA4-3′UTR-Mut. Furthermore, miR-29c-3p-mimics suppressed the expression of CDCA4 protein, and the miR-29c-3p-inhibitor increased it remarkably. Therefore, there was a targeted regulatory relationship between miR-29c-3p and CDCA4. A cotransfection experiment demonstrated that after transfecting miR-29c-3p-mimics+sh-CDCA4 or miR-29c-3p-inhibitor+si-CDCA4 to M21 and C8161 cells, the biological functions of cells showed no significant difference compared with the miR-NC group. However, compared with the cells transfected with miR-29c-3p-mimics, the cells showed enhanced proliferation, migration, invasion, and weakened apoptosis, while compared with miR-29c-3p-inhibitor, all the results were reversed. So the targeted regulatory relationship between miR-29c-3p and CDCA4 was confirmed. Through the above tests, we initially proved that upregulation of miR-29c-3p inhibited CDCA4 expression, thus preventing malignant biological progress of MM. In the study by Wang et al., taurine-upregulated gene 1 (TUG1) regulates proliferation, invasion, and apoptosis of MM cells by mediating miR-29c-3p, suggesting that miR-29c-3p may be a therapeutic target in the pathological mechanism of MM [30]. Furthermore, Alderman and Yang [31] reported that CDCA4, targeted by miR-15a, regulates the proliferation, cycle, and migration of MM cells, suggesting that CDCA4 is also a potential novel therapeutic target for MM.

The apoptosis and EMT of MM cells are closely related to the malignant progression of tumors [32, 33], so studying these two biological processes would help us to further understand the regulatory mechanism of MM. Therefore, we measured the expression of apoptosis-related proteins (Bax, Caspase3, and Bcl-2) and EMT-related proteins (N-cadherin, vimentin, and E-cadherin) in MM cells under different transfection backgrounds. Bax and Caspase3 are well-known proapoptotic proteins, and Bcl-2 is an antiapoptotic protein, all of which are involved in the apoptosis mechanism of MM cells [34, 35]. N-cadherin, vimentin, and E-cadherin are important proteins involved in the EMT of MM cells. The decrease of N-cadherin and vimentin and the increase of E-cadherin generally portend the suppressed EMT, which is one of the positive manifestations of the inhibition of MM invasion and metastasis [36]. In our study, MM cells transfected with miR-29c-3p-mimcs or si-CDCA4 exhibited protein expression unfavorable to MM progression, that is, the expressions of Bax, Caspase3, and E-cadherin proteins were remarkably elevated and those of Bcl-2, N-cadherin, and vimentin were remarkably suppressed. However, miR-29c-3p-mimics+sh-CDCA4, miR-29c-3p-inhibitor+si-CDCA4, and miR-NC transfection induced little difference in the expression of related proteins. So it was inferred that upregulation of miR-29c-3p suppressed CDCA4 in a targeted manner, as well as hindered malignant progression of MM cells by promoting the antiapoptosis mechanism and inhibiting EMT of MM cells.

To sum up, miR-29c-3p hinders progression of MM through targeted inhibition of CDCA4. However, there is still room for improvement in this study. Firstly, it is necessary to analyze the relevant regulatory mechanisms in depth so as to investigate the potential mechanisms in this targeted relationship. Secondly, we should assess the value of sera miR-29c-3p and CDCA4 for predicting the efficacy in MM and find out whether there are dynamic changes in patients before and after treatment, thus exploring the potential clinical application value of the two.

## Figures and Tables

**Figure 1:** Expression and diagnostic value of sera miR-29c-3p and CDCA4. (a) Expression of serum miR-29c-3p in the MM group is remarkably lower than that in the normal group. (b) Expression of serum CDCA4 in the MM group is remarkably higher than that in the normal group. (c) AUC of miR-29c-3p and CDCA4 for diagnosing MM are 0.912 and 0.939, respectively. (d) Serum miR-29c-3p is closely negatively correlated with CDCA4 expression (*r* = −0.671, *P* < 0.001). Note: ^∗∗∗^*P* < 0.001.

**Figure 2:** Prognostic value of sera miR-29c-3p and CDCA4 in MM. (a) Low miR-29c-3p and high CDCA4 are significantly correlated with poor prognosis of MM patients. (b) AUC of sera miR-29c-3p and CDCA4 for predicting poor prognosis of MM are 0.830 and 0.842, respectively. (c) Low miR-29c-3p is significantly correlated with the lower 3-year OS of MM patients. (d) High CDCA4 is significantly correlated with the lower 3-year OS of MM patients. Note: ^∗∗∗^*P* < 0.001.

**Figure 3:** Effects of miR-29c-3p on biological functions of MM cells and EMT-related proteins. (a) miR-29c-3p is lowly expressed in MM cells, especially in M21 and C8161 cells. (b) Expression of miR-29c-3p is elevated markedly in cells transfected with miR-29c-3p-mimics. (c) Proliferation of cells transfected with miR-29c-3p-mimics is hindered markedly. (d) Migration of cells transfected with miR-29c-3p-mimics is hindered markedly. (e) Invasion of cells transfected with miR-29c-3p-mimics is hindered markedly. (f) Expression of Bcl-2 protein in the cells transfected with miR-29c-3p-mimics is remarkably suppressed, while those of Bax and Caspase3 proteins are remarkably elevated. Apoptosis of cells transfected with miR-29c-3p-mimics is significantly enhanced. The protein map and flow cytometry diagram are provided. (g) Expression of N-cadherin and vimentin proteins in the cells transfected with miR-29c-3p-mimics is remarkably suppressed, while that of E-cadherin protein is remarkably elevated. The protein map is provided. Note: ^∗^*P* < 0.05, ^∗∗^*P* < 0.01 vs. the miR-NC group or HFF cells; ^#^*P* < 0.05 vs. the miR-29c-3p-inhibitor group.

**Figure 4:** Effects of CDCA4 on biological functions of MM cells and EMT-related proteins. (a) CDCA4 is highly expressed in MM cells, especially in M21 and C8161 cells. (b) Expression of CDCA4 is suppressed markedly in cells transfected with si-CDCA4. (c) Proliferation of cells transfected with si-CDCA4 is hindered markedly. (d) Migration of cells transfected with si-CDCA4 is hindered markedly. (e) Invasion of cells transfected with si-CDCA4 is hindered markedly. (f) Expression of Bcl-2 protein in cells transfected with si-CDCA4 is remarkably suppressed, while those of Bax and Caspase3 proteins are remarkably elevated. Apoptosis of cells transfected with si-CDCA4 is significantly enhanced. The protein map and flow cytometry diagram are provided. (g) Expression of N-cadherin and vimentin proteins in the cells transfected with si-CDCA4 is remarkably suppressed, while that of E-cadherin protein is remarkably elevated. The protein map is provided. Note: ^∗^*P* < 0.05, ^∗∗^*P* < 0.01 vs. the miR-NC group or HFF cells; ^#^*P* < 0.05 vs. the miR-29c-3p-inhibitor group.

**Figure 5:** Detection of luciferase activity. (a) There are targeted binding loci between miR-29c-3p and CDCA4. (b) Relative luciferase activity-DLR assay. (c) Expression of CDCA4 protein in transfected M21 and C8161 cells. (d) Protein map. Note: ^∗∗^*P* < 0.01.

**Figure 6:** Cell cotransfection. (a) Cell proliferation after transfecting miR-29c-3p-mimics+sh-CDCA4. (b) Cell migration after transfecting miR-29c-3p-mimics+sh-CDCA4. (c) Cell invasion after transfecting miR-29c-3p-mimics+sh-CDCA4. (d) Expression of Bax, Caspase3, Bcl-2, and other apoptosis-related proteins and apoptosis after transfecting miR-29c-3p-mimics+sh-CDCA4. The protein map and flow cytometry diagram are provided. (e) Expression of EMT-related proteins after transfecting miR-29c-3p-mimics+sh-CDCA4. The protein map is provided. Note: ^∗^*P* < 0.05, ^∗∗^*P* < 0.01 vs. the miR-NC group or HFF cells; ^#^*P* < 0.05 vs. the miR-29c-3p-inhibitor group.

**Table 1:** Association between miR-29c-3p, CDCA4, and pathological data (*n* (%), mean ± SD).

Factor	*n* = 59	miR-29c-3p	*T*	*P*	CDCA4	*T*	*P*
Sex			0.824	0.414		0.569	0.572
Male	33	0.83 ± 0.24			2.18 ± 0.36		
Female	26	0.88 ± 0.22			2.13 ± 0.30		
Age (years)			0.893	0.376		0.768	0.446
<60	31	0.86 ± 0.20			2.11 ± 0.29		
≥60	28	0.81 ± 0.23			2.17 ± 0.31		
T staging			2.885	0.006		1.903	0.062
T2/T3	45	0.94 ± 0.27			2.06 ± 0.31		
T4	14	0.72 ± 0.16			2.23 ± 0.22		
N staging			3.112	0.003		3.033	0.004
N0	17	0.96 ± 0.19			2.04 ± 0.20		
N1	42	0.75 ± 0.25			2.26 ± 0.27		
M staging			3.178	0.002		3.265	0.002
M0	48	0.98 ± 0.27			2.02 ± 0.22		
M1	11	0.71 ± 0.16			2.25 ± 0.16		
Tumor diameter (cm)			3.529	<0.001		2.970	0.004
<5	34	0.95 ± 0.23			2.05 ± 0.19		
≥5	25	0.74 ± 0.22			2.22 ± 0.25		
Pathological differentiation			3.965	<0.001		3.246	0.002
Poorly differentiated	35	0.70 ± 0.24			2.28 ± 0.36		
Moderately and highly differentiated	24	0.94 ± 0.21			1.99 ± 0.30		

**Table 2:** Univariate and multivariate Cox regression analyses.

Indicator	Univariate		Multivariate	
	HR (95% CI)	*P*	HR (95% CI)	*P*
Sex	1.209 (0.789-2.173)	0.216		
Age	1.105 (0.890-1.542)	0.099		
T staging	1.957 (2.016-2.163)	0.016	1.646 (1.446-2.971)	0.012
N staging	3.869 (1.485-3.420)	<0.001	3.365 (2.329-4.122)	0.001
M staging	2.224 (1.196-3.775)	0.009	2.531 (0.817-3.924)	0.002
Tumor diameter	1.563 (1.017-2.491)	0.043	1.768 (0.465-2.354)	0.001
Pathological differentiation	2.832 (1.334-11.365)	0.001	3.665 (0.845-9.954)	0.005
miR-29c-3p	7.036 (1.564-9.254)	0.004	6.174 (1.341-28.315)	0.020
CDCA4	5.111 (1.021-21.708)	0.011	7.033 (1.562-9.246)	0.003

## Data Availability

All the raw data could be accessed by contacting the corresponding author on reasonable request.
